The article "Wetland Ecotourism Development Using Deep Learning and Grey Clustering Algorithm from the Perspective of Sustainable Development" was published in 2022. Journal: J Environ Public Health.

# Wetland Ecotourism Development Using Deep Learning and Grey Clustering Algorithm from the Perspective of Sustainable Development

**DOI:** 10.1155/2022/1040999

**Published:** 2022-08-04

**Authors:** Bintao Shao, Longtao Chen, Nian Xing

**Affiliations:** ^1^School of Economics and Management, Shihezi University, Shihezi, Xinjiang 832000, China; ^2^School of International Economy and Trade, Wuxi University, Wuxi 214105, China; ^3^School of Journalism and Communication, Sichuan International Studies University, Chongqing 400031, China

## Abstract

The purpose is to promote the sustainable development of wetland ecotourism in China and plan the passenger flow in different tourism periods. This work selects Zhangye Heihe wetland ecotourism spot as the research object. Firstly, the two single wetland ecotourism Demand Prediction Models (DPMs) are proposed based on the time series of the optimized Fuzzy Clustering Algorithm (FCA), grey theory, and the Markov Chain Method. The proposed wetland ecotourism DPM simulates and predicts the ecotourism passenger flow of wetland-scenic spots and verifies the maximum passenger flow. Then, a hybrid model combining the above two single models is proposed, namely, the wetland ecotourism DPM based on an optimized fuzzy grey clustering algorithm. Further, the proposed three models predict the passenger flow in wetland ecotourism spots from 2015 to 2019. A wetland Water Quality Evaluation (WQE) model based on Deep Learning Backpropagation Neural Network (Deep Learning (DL) BPNN) is proposed to evaluate the water quality in different water periods. The results show that the hybrid model's Mean Absolute Percentage Error (MAPE) and Root Mean Square Error (RMSE) are 1.25% and 0.2532. By comparison, for two single models, the MAPE is 11.67% and 1.45%, respectively, and the RMSE is 0.2526 and 0.1652, respectively. Therefore, the mixed hybrid has the highest accuracy and stability. The water quality of the scenic spot in the wet season is obviously better than that in the dry season and flat season. It is suggested that the natural environmental factors, such as water quality and passenger flow in different periods, should be considered when formulating ecotourism development strategies.

## 1. Introduction

Wetland is probably the best place for leisure tourism and an ecosystem with various resources for human existence. Thus, wetlands are considered to be the most effective and diversified ecological system in nature, upon which human survival and development depend. Wetlands are also the foundation for hydraulic engineering and water civilization [1, 2]. With the expansion of the global population, particularly the overwhelming number of tourists, and reckless exploitation, the ecological systems, such as wetlands, are being damaged and quickly disappearing. It only serves short-term and unsustainable social development. Meanwhile, the general population does not clearly know the wetland ecosystem, resulting in unreasonable use, large-scale destruction, and intentional waste of wetland resources [3]. The diminishing wetlands and their ecological functions threaten the fragile wetland biological systems, thereby affecting the human species' socioeconomic advancement [4]. Therefore, in response to the central government's sustainable development policies in China [5], it is urgent to efficiently plan the development of wetland ecotourism.

The tourism market is driven by tourism demand which is the critical profitability factor. Under inaccurate estimation of tourism demand, tourism supply may exceed demand, resulting in waste of resources. Hence, tourism investment and development policies should be formulated based on an accurate estimation of tourism demand [6]. Bose and Mali found an alternative solution for seasonal tourism demand estimation through the analysis of the multisequence structure time series method based on new data restorage technology [7]. Jahani et al. analyzed the tourism impact evaluation model and accurately estimated the tourism pressure through the change in vegetation density [8]. Currently, the tourism DPM is inaccurate and unstable. To sum up, scholars have studied tourism demand from many aspects, which is paramount for predicting and mining tourism demand. However, the prediction of passenger flow from the aspect of wetland WQE in ecological scenic spots is not involved in the above research. Thus, there are also some deficiencies in the above research methods. In the development of information technology, Deep Learning (DL) and Grey Clustering Algorithms (GCAs) gather some observation indexes or observation objects into several definable categories according to the grey incidence matrix or the whitening weight function grey number. According to different clustering objects, it can be divided into grey correlation clustering and grey-whitening weight function clustering. The grey model can be combined with wetland WQE and existing mathematical and statistical methods for modeling and simulation. Thus, the grey model is more prevalent in tourism development and pedestrian flow prediction.

This work puts forward the wetland ecotourism DPM based on grey theory, cluster analysis, and Markov Chain Method (MCM). The proposed wetland ecotourism DPM can estimate the passenger flow of scenic wetland spots in different years. The main innovation is to monitor the water quality of wetland ecotourism using the Deep Learning Backpropagation Neural Network (DL BPNN). It simulates and predicts the tourism demand based on the time series of optimized GCA and the water quality rating of wetland ecotourism spots. The finding provides a practical basis for China's efficient and rapid development of wetland ecotourism spots.

## 2. Methodology

### 2.1. Tourism DPM Using Time Series Based on Optimized FCA

Model construction: The existing fuzzy time series generally includes four aspects. The first is the definition and domain division. The second is to fuzzify historical data. The third is to establish fuzzy logic relations and get the fuzzy relation group. The fourth is to calculate the fuzzy relation and produce the corresponding results [9, 10]. Here, based on the analysis of the existing algorithms, the K-means clustering algorithm can optimize the domain division and establish the fuzzy logic relation for estimation using the automatic clustering algorithm [11]. The specific algorithm steps are as follows.

**Step 1 .**

Data sorting: The sample data sequence is rearranged. The processed wetland ecotourism's demand data sequence *M* can be expressed as follows:

(1) $$\begin{array}{c} M=m_{1},m_{2},\ldots ,m_{i},\ldots m_{n}. \end{array}$$

**Step 2 .**

The domain of the observed value is defined, and the interval is divided. The maximum *m*_*n*_ and minimum *m*_1_ in the sequence are found in equation (1). Suppose that the domain is H, then H can be defined as follows:

(2) $$\begin{array}{c} H=\left[m_{1}-P_{1},m_{n}-P_{2}\right]. \end{array}$$

In equation (2), *P*_1_ and *P*_2_ represent the required random positive numbers. Based on the characteristic values of the data sequence, the integral parts of the number are generally selected. Firstly, SPSS26.0 can call the K-means algorithm to cluster the *M* sequence to obtain *k* cluster centers. Then, the medians of two adjacent *K* centers are calculated successively to obtain *K*−1 values and introduced into the domain *H* to obtain *K* initial intervals (*H*_1_, *H*_2_, *K*, and *H*_*k*_). The absolute value of the difference between two adjacent data in sequence *M* and the mean of the absolute value is calculated. Then half of the mean is regarded as the maximum allowable distance of the interval. These values are introduced into *K* initial intervals. The initial interval is divided twice. The length of each interval is different because the distribution of the data in the domain is not uniform, and the clustering results can divide the subintervals. Compared with the equal domain division, the distribution of the data structure can be better reflected, improving the estimation accuracy. Finally, the historical data are introduced into the corresponding interval. Each set of historical data corresponds to an interval.

**Step 3 .**

The data is fuzzified, and the logical relation is established. The fuzzy set *Q*_*i*_ is defined according to the interval obtained in step 2. The historical data is fuzzified according to the following:

(3) $$\begin{array}{c} \left\{\begin{array}{c} Q_{1}=\frac{f_{11}}{H_{1}}+\frac{f_{12}}{H_{2}}+\cdots +\frac{f_{1n}}{H_{n}}\\ Q_{2}=\frac{f_{21}}{H_{1}}+\frac{f_{22}}{H_{2}}+\cdots +\frac{f_{2n}}{H_{n}}\\ \cdots \\ Q_{n}=\frac{f_{n1}}{H_{1}}+\frac{f_{n2}}{H_{2}}+\cdots +\frac{f_{nn}}{H_{n}} \end{array}\right)\Rightarrow \\ \left\{\begin{array}{c} Q_{1}=\frac{1}{H_{1}}+\frac{0.5}{H_{2}}+\frac{0}{H_{3}}+\cdots +\frac{0}{H_{n}},\\ Q_{2}=\frac{0.5}{H_{1}}+\frac{1}{H_{2}}+\frac{0.5}{H_{3}}+\cdots +\frac{0}{H_{n}},\\ \cdots ,\\ Q_{n}=\frac{0}{H_{1}}+\frac{0}{H_{2}}+\cdots +\frac{0}{H_{n-1}}+\frac{1}{H_{n}}. \end{array}\right) \end{array}$$

After fuzzification, the fuzzy logic relation can be obtained, namely *Q*_*i*_⟶*Q*_*j*_ (if the *m*^th^ year corresponds to *Q*_*i*_, then the *m* + 1^th^ year belongs to *Q*_*j*_).

**Step 4 .**

Defuzzification and estimation. Here, the wetland ecotourism demand is estimated, and the mathematical expression can be expressed as follows:

(4) $$\begin{array}{c} U_{j}=\frac{\left(w+E\left[Q_{j}^{*}\right]\right)}{\left(R+1\right)}, \end{array}$$

(5) $$\begin{array}{c} \left\{\begin{array}{c} R_{i}=\left|\left|O_{i}-O_{i-1}\right|-\left|O_{i-1}-O_{i-2}\right|\right|,\\ X_{i}=O_{i}+\frac{R_{i}}{2},\\ XX_{i}=O_{i}-\frac{R_{i}}{2},\\ Y_{i}=O_{i}+R_{i},\\ YY_{i}=O_{i}-R_{i}, \end{array}\right) \end{array}$$

In equations (4) and (5), [*Q*_*j*_^*∗*^] denotes the interval *H*_*j*_ with a membership degree of 1 in fuzzy set *Q*_*j*_, *O*_*i*_ represents the actual data of the *m*^th^ year, and *U*_*j*_ stands for the estimated value of the *m* + 1^th^ year. If the third-order model is adopted, the data of the *m* + 1^th^ year are estimated through the data of the (*m* − 2)th, (*m* − 1)th, and *m*th years, and then each index is calculated through equation (5). Similarly, if the fourth-order model is adopted, it is so deduced.

**Step 5 .**

Model accuracy evaluation. Here, the model accuracy is estimated based on the MAPE and RMSE. The calculation process is shown as follows:

(6) $$\begin{array}{c} \text{MAPE}=\frac{\sum_{i=1}^{m}\left|\overset{\wedge }{y_{i}}-y_{i}\right|/y_{i}}{m}, \end{array}$$

(7) $$\begin{array}{c} \text{RMSE}=\sqrt{\frac{\sum_{i-1}^{m}{\left(\overset{\wedge }{y_{i}}-y_{i}\right)}^{2}}{m}}. \end{array}$$

In equations (6) and (7), $\overset{\cap }{y_{i}}$ represents the estimated value, *y*_*i*_ denotes the actual value, and *m* stands for the number of test data. The smaller the MAPE and RMSE are, the higher the estimation accuracy of the model is.

### 2.2. Tourism DPM Based on Fuzzy Grey Markov Chain

Data of the tourism system are uncertain, incomplete, dynamic, and limited, much in line with the characteristics of a grey system, so the grey system theory can estimate the tourism demand [12]. The deepening research of grey estimation theory suggests that the grey system estimation method shows less accuracy and precision due to the disorder of initial data [13]. Therefore, a new tourism DPM is proposed based on fuzzy grey theory and the MCM [14].

First, the grey theory is discussed. The subjects of grey system theory [15] are uncertain systems with partial information. Information generation and extraction can obtain valuable information to accurately describe and effectively control system operation behavior and evolution rules. Grey system theory is composed of a grey estimation model, grey clustering analysis, grey correlation analysis, grey decision-making method, and grey sequence operator, and the main technical contents include data processing and analysis, model construction, major problem decision, and development trend estimation. Estimation is to speculate and understand the future through past exploration. Grey estimation [16] processes the original data through grey system theory, establishes an estimation model, studies and discovers the system's development law, and scientifically and quantitatively estimates the future state and trend of the system.

The wetland ecotourism demand is a comprehensive random event of fuzziness and contingency. It is estimable with grey theory. Thus, the grey GM (1,1) model [17] is chosen for estimation, the basic grey system theory model. The basic idea is to establish an estimation model by transforming the original irregular sample data sequence to obtain a new and uniform data sequence. The modeling of the grey GM (1,1) model is as follows.

#### 2.2.1. Data are Preprocessed

Original data are mostly irregular and random and cannot construct the model directly, so the original data sequence should be preprocessed. If the original data sequence is *D*_0_, then the following equation can be obtained:

(8) $$\begin{array}{c} D_{0}=\left\{D_{0}\left(1\right),D_{0}\left(2\right),\ldots ,D_{0}\left(m\right)\right\}. \end{array}$$

Then, the original data are judged for modeling applicability as follows:

(9) $$\begin{array}{c} \alpha \left(k\right)=\frac{D_{0}\left(k-1\right)}{D_{0}\left(k\right)},\;k=2,3,\ldots ,M. \end{array}$$

In equation (9), if *α* (*k*) is covered, the original data sequence can be used for the estimation model. Otherwise, the original data sequence should be corrected to the allowable coverage. Then the corrected data sequence is used for modeling and estimation. Generally, the translation variation method is adopted.

(10) $$\begin{array}{c} Y_{0}\left(k\right)=D_{0}\left(k\right)+z,\;k=1,2,\ldots M. \end{array}$$

In equation (10), (*Y*_0_) represents the estimated value of modeling, and *z* is a constant. The new data sequences can be obtained through continuous cumulation based on the above operations.

#### 2.2.2. Matrix and Vector are Constructed

The new data sequence obtained through equation (11) improves the regularity of the original data sequence and reduces the randomness. With the increase of the cumulative number, the randomness weakens more. The cumulative matrix *G* and constant term vector *l* are constructed through equations (12) and (13) as follows:

(11) $$\begin{array}{c} G=\left[\begin{array}{cc} -\frac{\left(D_{1}\left(2\right)+D_{1}\left(1\right)\right)}{2} & 1\\ -\frac{\left(D_{1}\left(3\right)+D_{1}\left(2\right)\right)}{2} & 1\\ \cdots & \;\\ -\frac{D_{1}\left(n\right)+D_{1}\left(n-1\right)}{2} & 1 \end{array}\right], \end{array}$$

(12) $$\begin{array}{c} Y_{m}={\left(D_{0}\left(2\right),D_{0}\left(3\right),\ldots ,D_{0}\left(m\right)\right)}^{T}. \end{array}$$

In equation (13), *T* represents the time set.

Afterward, the basic form of the GM (1,1) model is constructed. Assume that the development coefficient is *h*, and the grey action is *f*, then equation (13) can be obtained through the LSM (Least Squares Method) as follows:

(13) $$\begin{array}{c} f=\frac{dD_{1}}{\text{d}t}+hD_{1},\\ \overset{\wedge }{h}=\left[\begin{array}{c} h\\ f \end{array}\right]={\left(F^{T}F\right)}^{-1}F^{T}Y_{m}. \end{array}$$

The estimation model can be obtained through the introduction of *h* and *f* into the time function, as follows:

(14) $$\begin{array}{c} \overset{\wedge }{D_{1}}\left(m+1\right)=\left(D_{0}\left(1\right)-\frac{f}{h}\right)e^{-hk}+\frac{f}{h},\;k=1,2,\ldots m. \end{array}$$

Equation (15) can be obtained through the derivation of $\overset{\wedge }{D_{1}}$ in equation (14) as follows:

(15) $$\begin{array}{c} \overset{\wedge }{D_{0}}\left(m\right)=\overset{\wedge }{D_{1}}\left(m+1\right)-\overset{\wedge }{D_{1}}\left(m\right). \end{array}$$

In equation (15), $\overset{\wedge }{D_{0}}\left(m\right)$ represents the estimated value.

#### 2.2.3. The MCM is Explained

The Markov estimation method can estimate the probability of events. According to the current situation, the developmental change in each future period can be estimated.

Let *T* = {0,1,2,...} be a random process. Let *R* be a state space, *R* = {1,2,3,...}, random positive integers *i*_1_, *i*_2_, and *i*_3_, nonnegative integers *o*_1_, *o*_2_, and *o*_3_, *o*1>*L* > *o*2>*o*3, and the correspondent state are *E*_*i*_2_+*i*_3__, *E*_*i*_2__, *E*_*o*_1__, *L*, *E*_*o*_2__, *E*_*o*_3__, then equation (16) can be obtained as follows:

(16) $$\begin{array}{c} S\left\{E\left(i_{2}+i_{3}\right)\right\}=P\left\{E\left(i_{2}+i_{3}\right)\right\}=E_{i_{2}+i_{3}}|E\left(i_{2}\right)=E_{i_{2}}. \end{array}$$

Specifically, {*X*(*t*), *t* ∈ *T*} is the Markov chain. Usually, S_*Ei*_(*i*_2_) is related to states *E*, *i*, and *i*_2_. Only when S_Ei_(*i*_2_) is not related to *i*_2_, the Markov chain will contain stationary transition probability.

Finally, the tourism DPM based on a fuzzy grey MCM is constructed. Since the traditional grey estimation model is suitable for objects with less data, less time, and less fluctuation, it can estimate the changing trend of the whole system [18]. The Markov chain can estimate a random local change and generate different-state estimated values, leading to large deviation and thereby affecting the final estimation accuracy [19].

The fuzzy grey MCM is based on the traditional GM (1,1) method, which combines the advantages of the MCM with fuzzy classification theory. The fuzzy classification method is used at the end of the estimation period; any sample data may belong to different categories with different adherences. When the sample is disturbed, the estimated value changes. The adherence of the corresponding state class will change, and this method can improve its anti-interference ability [20]. The modeling steps of the fuzzy grey Markov chain estimation model are as follows.

**Step 6 .**

Data processing. According to the principle of grey estimation, GM (1,1) is established to achieve a fitting estimation according to the method in Section 2. Then the traditional grey parameters *h* and *f* are solved based on the original data sequence to establish a grey estimation model.

**Step 7 .**

After the accuracy is tested out according to the method in Section 2.1, the state division and fuzzy classification are carried out. The relative residuals between the original data sequence and the estimated value of the grey model are used as the division standard, and the system state is divided to obtain the membership function of the fuzzy set, obtaining the fuzzy state vector.

**Step 8 .**

Model accuracy test. Here, the residual test method [21] can evaluate the accuracy of the constructed model. The residual sequence is obtained from the original sequence and estimation sequence of the model: *μ*0 = {*μ*0(1), *μ*0(2), *L*, *μ*0(*m*)}. Then, the relative error *ψ*i and the average relative error can be expressed in the following equations, respectively:

(17) $$\begin{array}{c} \psi_{i}=\frac{u_{0}\left(i\right)}{D_{0}\left(i\right)}*100\%, \end{array}$$

(18) $$\begin{array}{c} \bar{\psi }=\frac{1}{m}\sum_{i=1}^{m}\left|\psi \left(i\right)\right|*100\%. \end{array}$$

In equations (17) and (18), *D*_0_ represents the initial value of the original sequence, and *m* denotes the number of test values. When the mean relative error is less than a given value, in general, if $\bar{\psi }$ <0.2, the model passes the residual test, indicating that the model has high accuracy.

### 2.3. Wetland Ecotourism DPM Based on Optimized Fuzzy GCA

Currently, the domestic tourism DPM is singular, while many internal and external factors may affect the tourism demand. A singular DPM can only capture some main factors and is incomplete and not fully effective, resulting in low accuracy and low stability in the estimation results [22, 23]. The hybrid estimation method can improve the accuracy and stability of the estimation result by utilizing effective information from every single model. Here, the fuzzy grey MCM is combined with the time series model based on fuzzy clustering to form a hybrid wetland ecotourism DPM.

Consequently, two single models of sections 2.1, 2.2 are combined. Assume that the weighted vector in the hybrid DPM is the estimation accuracy a-*λ* of *m* estimation methods at time *t* arranged in order from large to small. *a*−*λ* is the subscribe of the *n*th largest estimation accuracy; then equation (19) can be obtained as follows:

(19) $$\begin{array}{c} f_{w}\left(\langle a_{1t},D_{1t}\rangle ,\ldots ,\langle a_{mt},D_{mt}\rangle \right)=\sum_{i=1}^{m}w_{i}D_{a-\lambda }. \end{array}$$

In equation (19), *f*_w_ denotes the hybrid estimation value, indicating that the hybrid DPM is only related to the estimation accuracy of the single estimation methods at a given time point. Then, the hybrid DPM based on the minimum sum of squares of errors is expressed as follows:

(20) $$\begin{array}{c} \min R\left(w\right)=\sum_{i=1}^{m}\sum_{j=1}^{m}w_{i}w_{j}\left(\sum_{t=1}^{n}e_{a-i\lambda }e_{a-j\lambda }\right). \end{array}$$

In equation (20), ∑_*i*=1_^*m*^*w*_*i*_=1,  *w*_*i*_ ≥ 0,  *i*=1,2,…*m*, and *R* represents the sum of squares of the total error. Let $\bar{g_{1}}\left(T\right)=1/T\sum_{t=1}^{T-1}g_{i}\left(n-t\right),\;T=1,2,\ldots ,n$, and $\bar{g_{1}}\left(T\right)$ denotes the mean estimation accuracy from time *T* to *m*. The larger the value is, the higher the accuracy of the hybrid model is.

### 2.4. WQE of Wetland Based on BPNN

Backpropagation Neural Network (BPNN) is a multilayer feedforward Deep Learning Neural Network (DLNN) trained by the error Backpropagation (BP) algorithm. It has wide applications [24]. BPNN has the ability of arbitrary complex pattern classification and excellent multidimensional function mapping. Thus, it can solve problems that simple sensors cannot solve, such as the XOR problem [25]. BPNN comprises the input, hidden, and output layers. Specifically, the input layer represents the input of data elements. The hidden layer transmits signals between the input layer and the output layer. The output layer is responsible for the transfer and output of signal elements, as shown in Figure 1.

Essentially, the BP algorithm calculates the minimum object function (network error square) through the gradient descent method [26]. Assume that the input layer sample set *U* contains *m* training samples (vectors), and the index number of each sample is *n*. Assume that the training input is *I*, the output result is *Y*, the target result is *D*, and the weight is *p*. Then, the input of the *i*^th^ neuron in the first hidden layer is the weight product between the input layer and the first layer, as calculated through the following:

(21) $$\begin{array}{c} H_{1}^{i}=\sum_{n=1}^{n}p_{n}U_{Xn}. \end{array}$$

In equation (21), *U*_*xn*_ represents the *X*^th^ sample input vector.

The product of the output of the last hidden layer and the weight of the next hidden layer is the input of the next hidden layer. The results are transmitted in the network through the transfer function. The input of the output layer is output through the transfer function as the output of the *H*^th^ neuron [27], as expressed as follows:

(22) $$\begin{array}{c} Y_{D}^{D}=f\left(\sum_{b=1}^{B}p_{bp}Y_{b}^{B}\right). \end{array}$$

In equation (22), *Y* represents the output marker, *B* denotes the number of neurons in the final hidden layer, and *b* stands for the *b*^th^ neuron.

### 2.5. Model Parameters' Design

1. Here, the tourism number in Zhangye Heihe wetland from 2015 to 2019 are taken as the sample [from CSY (China Statistical Yearbook)]. The statistics are shown in Table 1.
2. Matrix Laboratory (MATLAB) can calculate the optimal weight coefficient of wetland ecotourism DPM based on optimized fuzzy GCA: *w*_1_ = 1, *w*_2_ = 0.
3. According to the standard water quality rating in the Environmental Quality Standard for Surface Water, the wetland WQE BPNN is trained. The output values of standard class I, II, III, III, IV, and V water quality are 0.1, 0.3, 0.5, 0.7, and 0.9, respectively. Here, ten water samples are randomly selected from Zhangye Heihe's wetland-scenic spot as BPNN's learning samples.

## 3. Results and Discussion

### 3.1. Results of the Tourism Demand Estimation Using Time Series Based on Optimized FCA

The fuzzy logical relation is obtained through the model calculation for the original data sequence of the number of tourists in the scenic area of Zhangye Heihe wetland from 2015 to 2019, as shown in Table 2.

Then, the number of wetland ecotourism in 2015–2019 is estimated, and the fitting estimation graph is shown in Figure 2.

Figure 2 illustrates that the actual tourism population from 2015 to 2019 is 16 million, 20.10 million, 25.99 million, 30 million, and 36.12 million, respectively. In contrast, the estimated number are 15.6 million, 19.95 million, 25.75 million, 29.68 million, and 35.96 million, respectively. The estimation errors are 400,000, 150,000, 240,000, 320,000, and 160,000, respectively. Thus, the estimability of the improved fuzzy time series model is good, and the error is small, indicating that the estimated value of the model is consistent with the actual situation.

Then, the improved fuzzy time series model is compared with relevant models in the field regarding their accuracy, as shown in Figure 3.

Figure 3 demonstrates that the MAPE of the optimized fuzzy time series model is small, only 1.45%, and the RMSE is 0.2532. Compared with model *M*_2_, the estimation accuracy has been greatly improved. Compared with model *M*_1_, their estimation accuracy is basically the same. However, the research model has strong estimation accuracy while simplifying the calculation process.

### 3.2. Wetland Ecotourism Demand Estimation Based on Fuzzy Grey MCM

According to the number of tourists in the scenic area of Zhang Ye Heihe wetland from 2015 to 2019, the GM (1,1) model simulation data are tested. The results are shown in Figure 4.

Figure 4 displays that the relative error between the actual value and the estimated value of the model is less than 8%, and the mean relative error is less than 0.2. The estimation accuracy of the model is 95.8%, indicating that the model has passed the residual test. The posterior variance of the model is less than 0.35, and the minimum error probability is greater than 0.95, indicating that the model has high accuracy. However, the relative error between the estimated value and the actual value of the model is greater than 5%, so the accuracy of the model estimation results needs to be further improved.

The estimated value of the model corrected through the MCM is shown in Figure 5.

Figure 5 implies that the relative error of the corrected fuzzy grey Markov chain estimation model is much smaller than that of the original grey theory model. The mean (1,1) relative error of the original grey GM model is 3.5%, and the mean relative error of the fuzzy Markov chain estimation model is 2.01%. Meanwhile, the maximum relative error of the corrected estimation results is less than 3.8%, which is about 2.9% lower than the maximum relative error of the original model. The estimation results of the corrected model are closer to the actual value, the fluctuation is small, and the overall accuracy of the estimation is greatly improved.

### 3.3. Estimation Results of Wetland Ecotourism Demand Based on Optimized Fuzzy GCA

A comparison of the estimated results of the three models is shown in Figure 6.

Figure 6 shows that the wetland ecotourism DPM based on the optimized fuzzy GCA (the hybrid model) has obtained more stable results, less estimation error, and higher accuracy. The MAPE of the overall estimation is 1.19%, while the corresponding values estimated by the two separate models are 1.45% and 2.01%, respectively. Besides, the RMSE of the hybrid DPM is the smallest of the three models. Thus, the hybrid DPM has better estimate ability, overcomes the estimation defects of a single model, and improves the accuracy and stability of estimation.

### 3.4. WQE Results of Zhangye Heihe Wetland Based on DL BPNN

BPNN WQE model for Zhangye Heihe wetland in dry season WQE results is shown in Figure 7.

Figure 7 suggests that the water quality of the wetland-scenic spot in the dry season is mostly maintained at level II. Only two monitoring points are at level III, and two monitoring points are at level IV. The output value of BPNN is between 0.3 and 0.8, and the lower the output value is, the better the water quality of the monitoring point is.

The WQE results of Zhangye Heihe wetland in level season based on the BPNN model are shown in Figure 8.

Figure 8 suggests that the water quality of half of the wetland-scenic spots is maintained at level II, and the other half is maintained at level III during the level season. The output value of BPNN is between 0.2 and 0.55. The lower the output value is, the better the water quality of the monitoring point is. In the level season, the quantity of water increases, and the water quality improves significantly.

The WQE results of Zhangye Heihe wetland in the wet season based on the BPNN model are shown in Figure 9.

Figure 9 illustrates that the water quality of six monitoring points in the wetland-scenic spot is maintained at level II in the wet season. Two points are at level III, and another two points are at Level I. The output value of BPNN is between 0.1 and 0.5, indicating that the water quantity and water quality of the wetland-scenic spot are greatly increased in the wet period. Hence, the scenic area of the Zhangye Heihe wetland is suitable for tourism during the wet season. During this time, the water quality is high, the climate is pleasant, and the passenger flow will increase.

## 4. Conclusion

Under the background of the rapid development of information technology, this work aims to develop and plan wetland ecotourism scientifically. Two single models are proposed using the time series of optimized FCA and the fuzzy grey MCM. The research implements the prediction model by optimizing the fuzzy GCA, and the feasibility of the research method has been verified. Then, based on the optimized fuzzy GCA, a hybrid wetland ecotourism DPM is proposed by combining two single models. The passenger flow in the Heihe wetland-scenic spot of Zhangye, from 2015 to 2019 is predicted. Further, a WQE model of wetland ecotourism spot based on DL BPNN is proposed to monitor the water quality in different water periods. The estimation accuracy of the hybrid model is higher than that of every two single models. Therefore, the hybrid DPM has better estimability, overcomes the estimation defects of a single model, and improves the accuracy and stability of estimation. The water quality of the ecotourism spots in the wet season is significantly better than that in the dry and flat seasons. This suggests that the tourism department should optimize the development planning according to the wetland-scenic spot's passenger flow and ecological environment to improve ecotourism economic benefits. Lastly, there are some deficiencies in this work. Mainly, the range and size of samples are relatively narrow. There are many wetland-scenic spots in China. However, only one wetland ecotourism spot is selected for the experiment. Meanwhile, there are few monitoring points for WQE, resulting in the low accuracy of the prediction model. The later research plan will expand the selection range of sample data and select more wetland ecotourism spots to verify the model.

## Figures and Tables

**Figure 1:** structure of BPNN.

**Figure 2:** Comparison of estimated and actual tourism population in Zhangye Heihe wetland from 2015 to 2019.

**Figure 3:** Errors of different models (*M*) the proposed optimization model *M*_1_: Model 1 in the field *M*_2_: Model 2 in this field).

**Figure 4:** GM (1,1) model simulation results.

**Figure 5:** Estimation results after model correction.

**Figure 6:** Comparison of estimation results of wetland ecotourism number of different models (a) comparison of the estimated number and the actual number of three models (b) MAPE and RMSE index values estimated by three models 1: Wetland ecotourism DPM of time series based on optimized FCA 2: Wetland ecotourism DPM based on fuzzy grey MCM 3: DPM for wetland ecotourism based on optimized fuzzy GCA).

**Figure 7:** Evaluation results of water quality of Heihe wetland in Zhangye in the dry season.

**Figure 8:** WQE results of Heihe wetland in Zhangye during the level season.

**Figure 9:** WQE results of Heihe wetland in Zhangye during the wet season.

**Table 1:** Tourism Number of Zhangye Heihe wetland in 2015–2019.

Year	The actual number of tourists (ten thousand)
2015	1,600
2016	2,010
2017	2599
2018	3,000
2019	3,612

**Table 2:** Fuzzy relation table.

Year	The actual number of tourists (ten thousand)	The fuzzified number of people
2015	1,600	*Q *_1_
2016	2,010	*Q *_2_
2017	2,599	*Q *_3_
2018	3,000	*Q *_4_
2019	3,612	*Q *_5_

## Data Availability

The raw data supporting the conclusions of this article can be obtained from the corresponding author upon request.
